The article "Chalcones: The flavonoid derivatives synthesis, characterization, their antioxidant and in vitro/in vivo antidiabetic potentials" was published in 2023. Journal: Heliyon.

# Chalcones: The flavonoid derivatives synthesis, characterization, their antioxidant and in vitro/in vivo antidiabetic potentials

**DOI:** 10.1016/j.heliyon.2023.e22546

**Published:** 2023-11-18

**Authors:** Jalal Uddin, Syed Wadood Ali Shah, Muhammad Zahoor, Riaz Ullah, Amal Alotaibi

**Affiliations:** a Department of Biochemistry, University of Malakand, Chakdara 18800, Pakistan; b Department of Pharmacy, University of Malakand, Chakdara 18800, Pakistan; c Medicinal Aromatic and Poisonous Plants Research Center, Department of Pharmacognosy, College of Pharmacy, King Saud University, Riyadh 11451, Saudi Arabia; d Department of Basic Sciences, College of Medicine, Princess Nourah Bint Abdulrahman University. Riyadh 11671, Saudi Arabia

**Keywords:** Chalcones, Diabetes, Antioxidant, Alpha glucosidase, DPPH

## Abstract

Chalcones (designated **JA1**, **JA2** and **JA3)** were prepared from aromatic aldehyde and acetophenone which were then characterized using various spectroscopic techniques. The antioxidant potential of synthesized compounds was evaluated against DPPH free radical whereas the antidiabetic potential was determined against alpha glucosidase. Further the antidiabetic potential of the synthesized compounds was evaluated in rat model which were given orally experimental animals in doses 10 and 20 mg/kg body weight. The blood biochemical parameters like total cholesterol, triglycerides, alanine phosphatase, serum glutamic pyruvic transaminase, serum glutamic oxaloacetic transaminase, serum creatinine, HDL, and LDL levels were determined using commercially available kits. The antioxidant potential was found high for **JA3** followed by **JA2** with IC_50_ value of 64.02 ± 1.47 μg/ml whereas against alpha glucosidase again the same compound with IC_50_ of 63.04 μg/ml exhibited highest inhibitory potential. The blood glucose level was brought to almost normal level (126.88 and 119.13 mg/dl at 10 and 20 mg/kg body weight) in diabetic rats (induced by STZ) by compound **JA3** at the tested doses in comparison to acarbose at day 28th. The blood biochemical parameters were normalized in diabetic rats by compound **JA3** compared with diabetic control group. Based on the results **JA3** should be considered as effective antioxidant and antidiabetic drug candidate.

## 1 Introduction

Diabetes mellitus is a group of related metabolic diseases with high level of glucose in the blood. It not only brings irregularities in carbohydrate metabolism but also adversely affect the protein and fat metabolism. Diabetes mellitus may cause a long-lasting neuropathic, microvascular and macrovascular problems [1]. Type 1 diabetes mellitus (T1DM) occurs due to the destruction of the beta cells of pancreas leading to the deficiency of insulin. Approximately 5–10 % cases reported around the globe are of the T1DM [2]. Type 2 diabetes mellitus is categorized by symptoms like reduced insulin secretion, non-functioning of the beta cell of pancreas, reduction in the mass of the beta cells and failure in the progression of the beta cells. Resistance to insulin occurs due to the extreme production of hepatic glucose, reduction in the uptake of glucose by skeletal muscles, high production of free fatty acid, and increased lipolysis. To normalize the glucose level, glucagon is secreted in a large quantity. T2DM may leads to nephropathy, retinopathy and neuropathy which are the microvascular complications whereas the macrovascular problems are manifested as peripheral vascular diseases and heart diseases. About 90 % cases reported are of the T2DM [3]. Another type of diabetes mellitus which occur in the pregnancy and in the last phase of the gestational period is referred to as the gestational diabetes mellitus [4].

The article "Chalcones: The flavonoid derivatives synthesis, characterization, their antioxidant and in vitro/in vivo antidiabetic potentials" was published in 2023. Journal: Heliyon.

Meglitinide**,** thiazolidinedione, sulfonylureas, dipeptidyl peptidase 4 inhibitors, biguanides and sodium-glucose cotransporter inhibitors are the major groups of the antidiabetic drugs [5]. Apart from the mentioned groups certain plants or their phytochemicals have antidiabetic potentials e.g. from the *Galega officinalis* plants Biguanide, guanidine and galegine have been extracted which lowers the blood glucose level [6]. Exenatide and Liraglutide are the two GLP-1 receptor agonists. Resistance to the dipeptidyle peptidase 4 has been shown by these two drugs. Linagliptin, alogliptin, saxagliptin, and sitagliptin are DPP-4 inhibitors and are used to control high blood sugar in adults with type 2 diabetes. Sodium glucose cotransporter inhibitors (SGLT) includes dapagliflozin, empagliflozin and canagliflozin have been reported as effective in treating DM [7]. Mostly, insulin administration is used to lower blood glucose level in DM [8]. The two important drugs in the class of meglitinides are the nateglinide and repaglinide are also effectively used in the treatment of Diabetes Mellitus [9]. Pioglitazone and rosiglitazone are the two drugs related to the class of thiazolidinedione and may be used to enhance the action of insulin [10]. Though the mentioned drugs are clinically proved antidiabetic drugs but none of them is 100 % efficient therefore, search for the most efficient drug is continued.

The word chalcone is derived from the Greek words Chalco meaning as bronze. Chalcones are organic compounds belonging to the family of flavonoid with a general formula of C_15_H_12_O [11]. Chalcones are chemically benzlidene acetophenone or benzaylacetophenone in which aromatic ring are connected to 3-carbon aliphatic chain. Different biological activities like antioxidant, anticancer, antimitotic and anti-inflammatory have been exhibited by the chalcones [12]. Due to the significant therapeutic potential of chalcones and their derivatives, they have also been used as antiprotozoal, antimicrobial, antihyperglycemic, anti-ulcerative, antitubercular, *anti*-HIV, anticonvulsant, antileishmanial, anticonvulsant, and antiviral agents [[13], [14], [15], [16]].

The article "Chalcones: The flavonoid derivatives synthesis, characterization, their antioxidant and in vitro/in vivo antidiabetic potentials" was published in 2023. Journal: Heliyon.

Herein we have tried to devise chalcones, the synthetic compounds to treat hyperglycemic conditions brought about by streptozotocin in rats used as animal model. The synthesized compounds designated as **JA1**, **JA2** and **JA3** were characterized by FTIR and HNMR techniques which were then used for in vitro evaluation of antioxidant and antidiabetic potentials respectively against DPPH and glucosidase markers. The compounds were then orally given to different groups of diabetic rats. The lipid profile, acute toxicity and blood biochemical parameters of experimental animal were also monitored.

## 2 Material and method

### 2.1 Chemical and reagents

All the chemical used herein were of analytical grade and used without further purification. NaOH, HCl, 4-bromoacetophenone, 2-chlorobenzaldehyde, 3-chlorobenzaldehyde, 4-chlorobenzaldehyde etc. were purchased from Sigma Aldrich, Germany.

### 2.2 General method for the synthesis of chalcone

To synthesize the desired compounds, 4-bromoacetophenone was mixed with substituted benzaldehyde and NaOH in methanol for 24–72 h. The reaction progress was monitored through TLC. At the completion of reaction, the mixture contents were added to the crushed ice and washed with the help of 0.1 N HCl. The chalcones formed were obtained in the form of precipitate which were then filtered off to separate from reaction mixture. Recrystallization was used for the purification of the product and finally the product was dried in oven. The general scheme of synthesis is presented in Fig. 1.

**Fig. 1:** Schematic presentation of chalcone synthesis.

#### 2.2.1 Synthesis of (E)-1-(4-bromophenyl)-3-(2-chlorophenyl) prop-2-ene-1one (**JA1**)

To a solution of NaOH (40 %) and 2-chlorobenzaldehyde in methanol, 4-bromoacetophenone was added and stirred for 24–72 h maintained at ambient temperature whereas the reaction progress was monitored through TLC. At completion of reaction, the contents were added to the crushed ice and washed with the help 0.1 N HCL. The product in the form of precipitate was filtered and recrystallized to purify it further which was then dried in oven (Fig. 2).

The article "Chalcones: The flavonoid derivatives synthesis, characterization, their antioxidant and in vitro/in vivo antidiabetic potentials" was published in 2023. Journal: Heliyon.

**Fig. 2:** Synthesis of **JA1**.

#### 2.2.2 Synthesis of (E)-1-(4-bromophenyl)-3-(3-chlorophenyl) prop-2-ene-1one (**JA2**)

To a stirring solution containing NaOH (40 %) and 3-chlorobenzaldehyde in methanol, 4-bromoacetophenone was added and mixed for 24–72 h at room temperature (Fig. 3). The subsequent detail of experimentation was similar as mentioned in section 2.2.1.

**Fig. 3:** Synthesis of **JA2**.

#### 2.2.3 Synthesis of (E)-1-(4-bromophenyl)-3-(4-chlorophenyl) prop-2-ene-1one (**JA3**)

To a stirring solution of NaOH (40 %) and 4-chlorobenzaldehyde in methanol, 4-bromoacetophenone was added and maintained at room temperature for 72 h. The reaction in schematic form is shown in Fig. 4. The subsequent experimental procedure was similar as mentioned above.

**Fig. 4:** Synthesis of **JA3**.

### 2.3 Determination of free radical scavenging by the synthesized compounds (DPPH assay)

DPPH a synthetic free radical was used as a reaction marker in the evaluation of antioxidant activity of the synthesized compounds. Oxidized form of the DPPH when dissolve in methanol give a deep violet color. On gaining the electron from the antioxidant, DPPH is reduced and its color changes to yellow which is the principle of this assay. About 20 mg of DPPH was dissolved in 100 ml of methanol that was used as stock solution. About 3 ml of the stock solution was taken and its absorbance was adjusted as 0.7 at 515 nm which was referred to as control solution. Aluminum foil was used to covered the solution of DPPH that was then kept for 24 h in a dark place for the production of free radicals. The synthesized compounds stock solutions were prepared by dissolving 5 mg of each in the 5 ml of methanol. Several solutions with different concentration (62.5–1000 μg/ml) from the stock solution were then prepared through serial dilution. About 2 ml from each dilution were then taken and mixed with 3 ml DPPH stock solution. The solutions were then placed for 15 min in dark to ensure the required incubation criteria. Ascorbic acid was used as standard. For the calculation of percent inhibition of DPPH scavenging by the synthesized compounds, the formula as given below, was used:

(1) $$\%\text{Free}\;\text{radicals}\;\text{scavenging}\;\text{potential}=\frac{\text{Blank}\;\text{sample}\;\text{absorbance}-\text{sample}\;\text{absorbance}}{\text{Blank}\;\text{sample}\;\text{absorbance}}\times 100$$

### 2.4 Assessment of in-vitro α-glucosidase inhibitory activity

The synthesized compounds were subjected to α-glucosidase inhibitory activity by constituting the reaction mixture consisting of 20 μl α-glucosidase (0.5 unit/ml), 120 μl of 0.1 M phosphate buffer of pH 6.9 and 10 μl of Chalcones in different concentration which were then thoroughly mixed. A 96-well microreader plates was used and the mixture was kept in incubator for 15 min at 37 °C. About 20 μl of 5 mM *p*-nitrophenyl-α-d-glucopyranoside solution in 0.1 M phosphate buffer of pH 6.9 was added to the reaction mixture and again placed in an incubator at 37 °C for 15 min to initiate the enzymatic reaction. Absorbance of reaction mixture was recorded using micro plate reader at 405 nm. To stop the reaction progress at the time of measurement, sodium carbonate (80 μl, 0.2 M) was added to the mixture. Sample free reaction mixture was used as positive control and for achieving the background absorbance correction a blank solution without α-glucosidase was utilized. Acarbose was used as standard [17].

(2) $$\%\alpha -\text{Glucosidase}\;\text{Inhibition}=\frac{\text{control}\;\text{absorbance}-\text{sample}\;\text{absorbance}}{\text{control}\;\text{absorbance}}\times 100$$

The article "Chalcones: The flavonoid derivatives synthesis, characterization, their antioxidant and in vitro/in vivo antidiabetic potentials" was published in 2023. Journal: Heliyon.

### 2.5 Estimation of the IC_50_ value

With the help of Excel 2007, the concentration of the synthesized compounds at which 50 % inhibition was observed (IC_50_), were estimated from the inhibition percentages recorded against the compound's concentration.

### 2.6 In vivo studies

Mice (20–25 g, 5–7 weeks old) and rats (190–210 g, 6–8 weeks old were brought from the NIH Islamabad to the University of Malakand. The animals were kept in a daily light/dark (16/8) cycle at 25 °C±2. Throughout the experiment for the safety of the well beings of the animals the national and institutional procedures for the regulation of the ethic were taken into consideration. ARRIVED guidelines were followed during course of the experiments whereas ethical approval was taken from Ethical Committee of the Department of Pharmacy, University of Malakand, vide notification Pharm/EC-HEREF/10–31/36 following the 2008 animal bylaws.

#### 2.6.1 Acute toxicity study

For the determination of acute toxicity of chalcones, animals having weight in the range of 20–25 g were used. Animals were distributed in different groups with each group containing 4 animals. The test was conducted in two phases following the reported protocol with slight changes. In the first stage, Tween-80 (2 %) was given to the control group and chalcones were given to another groups orally as 1000, 2000 and 3000 mg/kg body weight respectively [18]. The dose of 2000 mg/kg body was found safe with no casualties therefore, it was established that the compounds in doses up to 200 mg/kg body weight (b.w) will be safe which was 1/10th of highest safe dose per guide lines of OCED. However, due to limited quantities of the compounds in hand we have used doses 10 and 20 mg/kg b. w.

The article "Chalcones: The flavonoid derivatives synthesis, characterization, their antioxidant and in vitro/in vivo antidiabetic potentials" was published in 2023. Journal: Heliyon.

##### 2.6.1.1 Oral glucose tolerance test

The oral glucose tolerance test (OGTT) of **JA1** to **JA3** was performed in overnight fasted normal rats that were divided into different groups (n = 8). Group 1 was administered with 2 % (w/v) Tween-80, Group 2 received glibenclamide, while the remaining groups received the respective doses of test compounds. After 30 min, the animals were fed with glucose (3 g/kg). Blood glucose level was estimated at 0, 30, 60, and 120 min of glucose administration using SD glucometer (ACCU-CHECK, Active blood glucose meter, Korea).

#### 2.6.2 Induction of diabetes

For the induction of diabetes, the animals (rats) were first fasted overnight. In 0.1 mol citrate buffer of 4.5 pH Streptozotocin was prepared freshly and given in a single dose of 50 mg/kg body weight via intraperitoneally. Animals with fasting blood glucose level greater than 200 mg/dl were selected as diabetic animals [19].

#### 2.6.3 Animals grouping and dosing

A total of 72 animals after diabetes induction were divided into nine groups, each containing eight animals (n = 8), comprising diabetic, normal control, test groups (**JA1** to **JA3**) treated with 10 and 20 mg/kg b. w whereas the standard drug in a dose of 0.5 mg/kg was administered to one group, to compare the obtained results of test compound with standard drug. Normal saline as vehicle was administered to animals in STZ diabetic groups and in control (normal) group. The treated animals received (**JA1** to **JA3**) p. o. at their respective doses (10 and 20 mg/kg b. w) for 4 weeks. The grouping details with doses are summarized in Table 1.

**Table 1:** Animals grouping and dosing.

Group	Treatment	Dose (mg)	Administration route
**Control**	**Normal saline**	10	Orally
**Diabetic**	**Normal saline**	10	Orally
**Diabetic**	**JA1**	10	Orally
**Diabetic**	**JA1**	20	Orally
**Diabetic**	**JA2**	10	Orally
**Diabetic**	**JA2**	20	Orally
**Diabetic**	**JA3**	10	Orally
**Diabetic**	**JA3**	20	Orally
**Diabetic**	**Standard (Glibenclamide)**	0.5	Orally

#### *2.6.4* *Ex-vivo* investigation of blood profile

At the end of the study (28th day), once the antidiabetic assay was finished, all the animals were humanely euthanized with isoflurane, and blood samples were taken to evaluate the biochemical parameters. Lipid profiles including total cholesterol (TC), triglycerides (TGs), high density lipoprotein (HDL), low density lipoprotein (LDL), alkaline phosphatase (ALP), and insulin level were determined [31].

### 2.7 Analysis of data

All values herein are expressed as mean ± SEM (n = 8). One way ANOVA followed by Dunnett's post hoc multiple comparison test have been applied to determine the values of P. *P˂0.05, **P˂0.01 and ***P˂0.001 as comparison of diabetic control group vs test samples and glibenclamide treated groups.

The article "Chalcones: The flavonoid derivatives synthesis, characterization, their antioxidant and in vitro/in vivo antidiabetic potentials" was published in 2023. Journal: Heliyon.

## 3 Results and discussion

### *3.1* *Spectral, synthesis detail and physical properties of (E)-1-(4-bromophenyl)-3-(2-chlorophenyl) prop-2-ene-1one* (**JA1**)

It is a light-yellow solid (74.5 %) with molecular formula C_15_H_10_BrClO, mp: 197.68 °C. ^1^HNMR (300 MHz, CDCl_3_) δ 6.70 (d, 1H), 7.38 (d, m,1H), 7.51 (m, 5H), 7.72–7.82 (m, 3H).

The synthesized compound has molecular weight 321.96 with creamy white appearance. The reaction yields 86 % with R. f. = 0.67 (ethyl acetate: n-hexane 1.5:3.5). The compound shows complete solubility in chloroform.

### *3.2* *Spectral, synthesis detail and physical properties of (E)-1-(4-bromophenyl)-3-(3-chlorophenyl) prop-2-ene-1one***(JA2)**

It is a white solid (69.2 %) with molecular formula C_15_H_10_BrClO, mp: 105–107 °C. ^1^HNMR (300 MHz, CDCl_3_) δ 3.25–3.33 (m, 1H), 7.16–7.28 (m, 2H), 7.42–7.47 (t, 1H), 7.60–7.63 (d, 2H), 7.80–7.83 (d, 2H), 8.01–8.03 (d, 1H), 8.11–8.13 (m, 1H).

Its molecular weight is 321.60 and is a creamy white powder with 89 % as reaction yield having R. f. = 0.71 (ethyl acetate: n-hexane 1.5:3.5). The compound is considerably soluble in chloroform.

### *3.3* *Spectral, synthesis detail and physical properties of (E)-1-(4-bromophenyl)-3-(4-chlorophenyl) prop-2-ene-1one***(JA3)**

It is a white yellowish crystalline substance (81.3 %) having molecular formula C_15_H_10_BrClO, mp:165–167 °C. ^1^HNMR (300 MHz, CDCl_3_) δ 7.40–7.49 (m, 3H), 7.58–7.61 (d, 2H),7.65–7.68 (d, 2H), 7.75–7.81 (d, 1H), 7.88–7.91 (d, 2H)

This compound was confirmed by FT-IR spectrum which showed strong absorption band at 1656 cm^−1^ indicating stretching frequency of carbonyl of the chalcone which is conjugated with (C=C) group. Another band appears at 1604 cm^−1^ for alkene.

^13^CNMR spectrum shows peaks at:76.55 ppm for the CDCl3 solvent, 190.77 ppm for the ketone group of chalcone, 120–128 ppm for the alkene group of chalcone CH=CH, and 129–143 ppm for the two aromatic rings. *m*/*z*:321.96(100 %), 319.96(77.3 %), 323.96(24.5 %), 322.96(16.4 %), 320.96(12.6 %), 324.96(3.9 %).

Its molecular weight is 321.60 having a creamy white appearance with 83 % yield. The compound shows substantial solubility in chloroform.

### 3.4 Antioxidant potential of synthesized chalcones

Table 2 shows the free radical scavenging effects of the synthesized compounds. It is evident from the table that the compound **JA3** has high free radical scavenging activity with IC_50_ 64.02 ± 1.47 μg/ml. The synthesized compounds **JA2** and **JA1** have also exhibited reasonable antioxidant activity having IC_50_ 65.80 ± 1.62 and 69.21 ± 1.51 respectively. All these three compounds contained benzene ring as their integral parts in their structures and can therefore, stabilizes the free radical singlet electron by resonance effect.

The article "Chalcones: The flavonoid derivatives synthesis, characterization, their antioxidant and in vitro/in vivo antidiabetic potentials" was published in 2023. Journal: Heliyon.

**Table 2:** Antioxidant activity of the synthesized Chalcones.

Sample	DPPH IC_50_ (μg/ml)
JA1	69.21 ± 1.51
JA2	65.80 ± 1.62
JA3	64.02 ± 1.47
**Ascorbic acid**	15.17 ± 1.04

Values expressed as mean ± SEM n = 3.

### 3.5 In vitro antidiabetic potential of chalcones

Alpha amylase and glucosidase are the key enzymes of carbohydrate metabolism in human body. In normal circumstances the feedback inhibition mechanism keeps the excessive or diminished enzymatic activities in control. However, diseased conditions this feedback control is affected and inhibitors from outside sources are then prescribed by the physicians to minimize the excessive enzymatic activity. Diabetes mellitus is a life-threatening disease and to keep it under control inhibitors of the mentioned enzymes are used as a strategy to treat it. Herein we have made an attempt to evaluate the compound synthesized for its antidiabetic potential. The results are summarized in Table 3 which is only restricted to alpha glucosidase inhibitory activity. The alpha glucosidase inhibitory potential in terms of IC_50_ for **JA1** is 85.11 ± 1.29 μg/ml, for **JA2** it is 97.24 ± 1.48 μg/ml, whereas for **JA3** it is 63.04 ± 1.17 μg/ml indicating it to be the most potent compound. The alpha glucosidase inhibitory activity of acarbose in terms of IC_50_ was 60.38 ± 1.22 μg/ml. Among the synthesized chalcone **JA3** was found to be the most potent compound because its results are quite near to the standard acarbose IC_50_ value. The alpha glucosidase inhibitory activity by compound **JA3** was promising and found to be the most potent in comparison to **JA1** and **JA2**. This potency may be attributed towards the chemical structure of **JA3** as it contains both bromine and chlorine groups at para position that makes the compound to be a potent antidiabetic agent. Similarly, in **JA1** and **JA2,** the bromine is present in the structures of both at para position while chlorine in **JA1** is at ortho and **JA2** at meta position making them as excellent candidates to be used as antidiabetic agent.

**Table 3:** Alpha glucosidase inhibitory activity.

Sample	Glucosidase IC_50_ (μg/mL)
JA1	**85.11 ± 1.29**
JA2	**97.24 ± 1.48**
JA3	**63.04 ± 1.17**
**Acarbose**	**60.38 ± 1.22**

Values expressed as mean ± SEM n = 3.

### 3.6 In vivo antidiabetic potentials of the synthesized compounds

#### 3.6.1 Effects on blood glucose in OGTT

From Table 4 it is evident that there are no noteworthy variations among normal control and treated group's blood glucose levels measured at 30, 60, 90 and 120 min after administration of compounds in tested doses. The **JA1**, **JA2** and **JA3** treated group level of glucose was found significantly lower after oral administration. The blood glucose level of the control group was 167.80 mg/dl after 60 min. **JA1** at a dose of 10 mg/kg b. w lowered the blood glucose level to 120.18 md/dl. Similarly, group 4 treated with **JA1** with a dose of 20 mg/kg b. w, the blood glucose level was lowered to 115.41 mg/dl. For group 5 treated with **JA2** at a dose of 10 mg/kg b. w the blood glucose level was lowered to 126.09 mg/dl whereas for group 6 treated with **JA2** at a dose of 20 mg/kg b. w the blood glucose level dropped to 124.19 mg/dl. The group 7 treated with **JA3** with a dose of 10 mg/kg b. w the blood glucose level was lowered to 118.20 mg/dl whereas in the case of group 8 treated with same compound at a high dose of 20 mg/kg b. w the blood glucose level was dropped down to 114.21 mg/dl. The group 9 treated with the Glibenclamide with a dose of 0.5 mg/kg b. w the blood glucose level was 109.76 mg/dl (a standard drug).

The article "Chalcones: The flavonoid derivatives synthesis, characterization, their antioxidant and in vitro/in vivo antidiabetic potentials" was published in 2023. Journal: Heliyon.

**Table 4:** Blood glucose level in mg/dL.

Groups/dose (mg/kg)		Blood glucose level (mg/dL)				
		0min	30 min	60 min	90 min	120 min
Control		108.09 ± 4.30	181.35 ± 4.39^!!!^	167.80 ± 4.21^!!!^	143.21 ± 4.38^!!!^	125.83 ± 3.98^!!!^
**JA1**	**10**	106.21 ± 4.61	124.71 ± 4.04*	120.18 ± 4.71*	117.21 ± 4.91*	115.18 ± 4.72
	**20**	104.10 ± 4.82	118.19 ± 4.61**	115.41 ± 4.69**	115.30 ± 4.70**	113.31 ± 4.66
**JA2**	**10**	106.41 ± 4.79	131.29 ± 4.71*	126.09 ± 4.67*	122.91 ± 4.61*	120.67 ± 4.57
	**20**	105.19 ± 4.68	127.37 ± 4.87*	124.19 ± 4.70*	121.08 ± 4.77*	118.03 ± 4.81
**JA3**	**10**	108.11 ± 4.77	120.39 ± 4.67*	118.20 ± 4.61**	114.91 ± 4.91**	112.91 ± 4.71
	**20**	106.76 ± 4.82	116.98 ± 4.71**	114.21 ± 4.66**	113.21 ± 4.42**	109.70 ± 4.86*
**Standard (Glibenclamide)**	**0.5**	107.21 ± 4.76	111.51 ± 4.86**	109.76 ± 4.97***	107.31 ± 4.61***	105.12 ± 4.70*

All values are expressed as mean ± SEM, n = 8. One way ANOVA after which Dunnett's post hoc multiple comparison test to determine the values of P. ^!!!^P˂0.001 as comparison of diabetic control group *vs* control group. *P˂0.05, **P˂0.01 and ***P˂0.001 as comparison of diabetic control group *vs* test samples and glibenclamide treated groups, using one way ANOVA followed by Dunnet comparison.

After 120 min time interval of administration, it was observed that the blood glucose level of the control group was 125.83 mg/dl. **JA1** at a dose of 10 mg/kg b. w dropped the blood glucose level to 115.18 mg/dl whereas for the highest tested dose of 20 mg/kg b. w the drop observed was 113.31 mg/dl. For **JA2** at a dose of 10 and 20 mg/kg b. w the reduction in blood glucose level was noted high (120.67 mg/dl and 118.03 mg/dl respectively). For **JA3** at doses of 10 and 20 mg/kg b. w the decrease in glucose observed was significant with blood glucose values of 112.91 mg/dl and 109.70 mg/dl respectively. For Glibenclamide treated group with a dose of 0.5 mg/kg b. w the blood glucose level noted was 105.12 mg/dl.

The article "Chalcones: The flavonoid derivatives synthesis, characterization, their antioxidant and in vitro/in vivo antidiabetic potentials" was published in 2023. Journal: Heliyon.

From the values of the decrease in the level of blood glucose it was noticed that among these compounds **JA3** showed the best inhibitory activity against glucosidase.

#### 3.6.2 Effect on blood glucose in STZ induced diabetes

From Table 5, it is clear that there is a significant decrease in the glucose level of diabetic groups as compared to **JA1**, **JA2** and **JA3** treated groups with doses of 10 and 20 mg/kg body weight at day 1st, 7th, 14th, 21st and 28th. The blood glucose level of the control group was 110.08 mg/dl at 14th day (falling in normal range as compared to diabetic group). For the diabetic control group, the level of blood glucose was found to be 443.20 mg/dl. The group treated with **JA1** with a dose of 10 mg/kg b. w the blood glucose level lowered to 235.69 md/dl in comparison to diabetic group animals. Similarly, for the group treated with high dose of the same compounds (20 mg/kg b. w) lowered the glucose level to 219.41 mg/dl signifying the mild antidiabetic activity of this compound. The group treated with **JA2** at a dose of 10 mg/kg b. w brought the blood glucose level to 241.70 mg/dl and for high tested dose it was brought to 229.91 mg/dl, clearly pointing towards the antidiabetic potential of the compound. The group treated with **JA3** at doses; 10 and 20 mg/kg b. w lowered the blood glucose level 206.65 mg/dl and 184.12 mg/dl respectively clarifying its high potency as antidiabetic agent as compared to other two compounds of the same series. The group treated with the Glibenclamide at a dose of 0.5 mg/kg b. w the blood glucose level was lowered to 155.46 mg/dl. The results described are of the 14th day treatment, therefore still the blood glucose levels are high as compared to control group which has been lowered further with progression of treatment.

**Table 5:** Blood glucose level in STZ induced diabetic rats (mg/dL).

Groups/dose (mg/kg)		Blood glucose level (mg/dL)				
		Day 1	Day 7	Day 14	Day 21	Day 28
**Normal control**		110.65 ± 4.81	108.41 ± 4.66	110.08 ± 4.80	103.87 ± 4.81	105.62 ± 4.96
**Diabetic control**		428.22 ± 4.81^!!!^	432.71 ± 4.96^!!!^	443.20 ± 5.91^!!!^	438.81 ± 4.94^!!!^	428.67 ± 4.90^!!!^
**JA1**	**10**	426.41 ± 4.69	314.71 ± 4.79*	235.69 ± 4.80*	181.12 ± 4.82*	152.67 ± 4.76*
	**20**	431.70 ± 5.10	301.39 ± 4.93*	219.41 ± 4.71*	159.03 ± 4.71**	134.89 ± 4.63**
**JA2**	**10**	433.91 ± 4.93	323.19 ± 4.68*	241.70 ± 4.84*	188.11 ± 4.81*	164.31 ± 4.77*
	**20**	428.22 ± 4.77	312.90 ± 4.71	229.91 ± 4.78*	162.40 ± 4.73**	142.60 ± 4.68**
**JA3**	**10**	437.41 ± 4.80	279.81 ± 4.67*	206.65 ± 4.89**	151.13 ± 4.80**	126.88 ± 4.90***
	**20**	431.62 ± 4.87	266.70 ± 4.80**	184.12 ± 4.83***	138.56 ± 4.69***	119.13 ± 4.71***
**Standard (Glibenclamide)**	**0.5**	434.88 ± 5.01	231.71 ± 4.71***	155.46 ± 4.71***	122.14 ± 4.61***	105.83 ± 4.67***

All values are expressed as mean ± SEM, n = 8. One way ANOVA after which Dunnett's post hoc multiple comparison test to determine the values of P. ^!!!^P˂0.001 as comparison of diabetic control group *vs* control group. *P˂0.05, **P˂0.01 and ***P˂0.001 as comparison of diabetic control group *vs* test samples and glibenclamide treated groups, using one way ANOVA followed by Dunnet comparison.

The article "Chalcones: The flavonoid derivatives synthesis, characterization, their antioxidant and in vitro/in vivo antidiabetic potentials" was published in 2023. Journal: Heliyon.

The blood glucose level lowering effect of compound **JA3** was promising and found to be the most potent in comparison to **JA1** and **JA2**. This potency may be attributed towards the chemical structure of **JA3** as it contains both bromine and chlorine containing groups at para position that makes the compound to be potent one. Similarly, in **JA1** and **JA2,** the bromine is present at para positions while chlorine in **JA1** is at ortho and **JA2** at meta position indicating the compounds to be used as antidiabetic agents.

With the progress of treatment, the blood glucose level was further normalized on 28th day of treatment as described below. The blood glucose level of the control group was 105.62 mg/dl at 28th day whereas for diabetic control group it was 428.67 mg/dl. The groups treated with **JA1** at the mentioned tested doses lowered the blood glucose level to 152.67 mg/dl and 134.89 mg/dl signifying that prolong treatment with this compound could normalize the blood glucose level in STZ diabetic rats. Similarly, groups administered with **JA2** caused, a reduction in blood glucose that was 164.31 mg/dl and 142.60 mg/dl at the tested doses respectively (Fig. 5) were noted. Groups getting the lower and high tested doses of **JA3** brought down the glucose level to 126.88 mg/dl and 119.13 mg/dl on 28th day of treatment, signifying compounds to be more potent than the rest of two synthesized compounds. The Glibenclamide with a dose of 0.5 mg/kg b. w totally normalized the level to 105.83 mg/dl, being the reported standard drug prescribed for the treatment of diabetes.

**Fig. 5:** Blood glucose level in STZ induced diabetic rats (mg/dL).

The article "Chalcones: The flavonoid derivatives synthesis, characterization, their antioxidant and in vitro/in vivo antidiabetic potentials" was published in 2023. Journal: Heliyon.

#### 3.6.3 Effect on body weight

Table 6 represents the effect of diabetes on body weight and its back recovery when treated with the synthesized compounds. A significant weight loss can be seen in the diabetic group animals. On the other hand; **JA1**, **JA2** and **JA3** groups has significantly helped in recovery of the weight loss in comparison to diabetic animals’ group. The weight of the control group was 199.08 g at 14th day of experiment whereas for diabetic group it was 180.31 g indicating a weight loss with STZ treatment. The weight of the **JA1** treated animals at 14th day with doses 10 and 20 mg/kg b. w was found to be 195.90 g and 196.80 g; quite near to normal control group animals. For the same interval of experimental cycle **JA2** has normalized the body weight to 196.31 and 194.17 g **JA3** with doses of 10 and 20 mg/kg b. w has normalized the weight to 196.68 and 197.72 g which very close to normal control group values. Glibenclamide with a dose of 0.5 mg/kg b. w, being a standard drug normalized the body weight to 194.98 g.

**Table 6:** Effect of synthesized compounds on body weight of diabetic animals.

Groups/dose (mg/kg)		Body weight (g)				
		Day 1	Day 7	Day 14	Day 21	Day 28
**Normal control**		197.51 ± 4.71	196.18 ± 4.89	199.08 ± 4.91	202.32 ± 4.76	198.66 ± 4.64
**Diabetic control**		198.64 ± 4.66	178.81 ± 4.88^!!^	180.31 ± 4.71^!!^	161.54 ± 4.59^!!!^	150.48 ± 4.80^!!!^
**Standard (Glibenclamide)**		200.91 ± 4.61	197.20 ± 4.79*	194.98 ± 4.81**	192.81 ± 4.68***	193.72 ± 4.77***
**JA1**	**10**	197.21 ± 4.88	198.76 ± 4.71*	195.90 ± 4.76*	187.60 ± 4.91*	184.57 ± 4.69**
	**20**	199.61 ± 4.62	197.61 ± 4.91*	196.87 ± 4.59*	187.07 ± 4.71*	183.50 ± 4.73***
**JA2**	**10**	196.31 ± 4.77	197.03 ± 4.73*	196.31 ± 4.91*	184.28 ± 4.55*	184.42 ± 4.61**
	**20**	197.80 ± 4.82	196.41 ± 4.93*	194.17 ± 4.63**	186.72 ± 4.80*	186.76 ± 4.69***
**JA3**	**10**	201.03 ± 4.71	198.92 ± 4.83*	196.68 ± 4.84*	185.39 ± 4.73*	187.40 ± 4.91**
	**20**	195.71 ± 4.88	197.38 ± 4.16*	197.72 ± 4.60*	190.90 ± 4.82*	191.68 ± 4.71**

All values are expressed as mean ± SEM, n = 8. One way ANOVA after which Dunnett's post hoc multiple comparison test to determine the values of P. ^!!!^P˂0.001 as comparison of diabetic control group *vs* control group. *P˂0.05, **P˂0.01 and ***P˂0.001 as comparison of diabetic control group *vs* test samples and glibenclamide treated groups, using one way ANOVA followed by Dunnet comparison.

The results recorded on 28th day as described below; it can be seen that normal group animals have an average weight of 198.66 g whereas the diabetic group has the average weight of 150.48 g showing that diabetes has caused a significant weight loss which has been normalized by the synthesized compounds as per given detail. **JA1** has brough improvement in weight at doses of 10 and 20 mg/kg body weight daily for 28 days (184.57 and 183.50 g respectively). Similarly, **JA2** at mentioned doses has brought the improvement of about 184.42 and 186.72 g. The groups treated with **JA3** at the mentioned doses has recovered the encountered weight loss (187.40 and 191.68 g respectively) which was more significant than other two compounds tested. The weights recorded for Glibenclamide group was 193.72 g.

The article "Chalcones: The flavonoid derivatives synthesis, characterization, their antioxidant and in vitro/in vivo antidiabetic potentials" was published in 2023. Journal: Heliyon.

### 3.7 Antihyperlipidemic effects in STZ diabetic rats

Table 7, Table 8 shows the levels of cholesterol (CH), High density Lipoprotein (HDL), Low Density Lipoprotein (LDL) and Triglycerides (TG) in different group animals. The level of triglycerides, cholesterol, low density lipoprotein in the diabetic group animals were quite high as compared normal group whereas a significant decrease was evident for HDL in diabetic group. The standard drug and synthesized compounds have normalized their values as per given details in the respective table. **JA1**, **JA2** and **JA3** in doses of 10 and 20 mg/kg b. w has lowered the level of CH, TG and LDL in STZ diabetic rats whereas at the same time they have enhanced the level of HDL at the administered doses. The individual effects on lipid profile parameters have been described per given detail.

**Table 7:** Effects of the synthesized compounds on levels of cholesterol and triglycerides.

Groups/dose mg/kg		Total CH (mg/dL)	TG (mg/dL)
Normal control		87.71 ± 4.51	**82.66 ± 2.41**
Diabetic control		182.79 ± 4.70^!!!^	**165.39 ± 2.88**^**!!!**^
Standard (Glibenclamide)		89.93 ± 4.59***	84.05 ± 2.48***
JA1	**10**	137.33 ± 4.61*	136.11 ± 1.98*
	**20**	120.71 ± 4.69***	121.15 ± 2.31**
JA2	**10**	145.39 ± 4.80*	138.70 ± 2.09*
	**20**	134.29 ± 4.79*	120.38 ± 2.48**
JA3	**10**	130.15 ± 4.82**	127.86 ± 2.50**
	20	110.09 ± 4.73***	101.49 ± 2.11***

All values are expressed as mean ± SEM, *n* = *8* (see Fig. 7). One way ANOVA after which Dunnett's post hoc multiple comparison test to determine the values of P. ^!!!^P˂0.001 as comparison of diabetic control group *vs* control group. *P˂0.05, **P˂0.01 and ***P˂0.001 as comparison of diabetic control group *vs* test samples and glibenclamide treated groups, using one way ANOVA followed by Dunnet comparison.

**Table 8:** Antihyperlipidemic effects of the synthesized compounds in STZ diabetic rats.

Groups/dose mg/kg		HDL (mg/dL)	LDL (mg/dL)
Normal control		50.19 ± 1.80	**36.87 ± 2.02**
Diabetic control		20.89 ± 1.77^!!!^	**133.69 ± 2.98**^**!!!**^
Standard (Glibenclamide)		48.10 ± 1.97**	39.88 ± 1.91***
JA1	**10**	36.71 ± 2.03*	82.83 ± 2.41*
	**20**	39.62 ± 1.88**	77.28 ± 2.39**
JA2	**10**	33.81 ± 2.01*	90.87 ± 3.09*
	**20**	35.94 ± 1.89*	78.31 ± 2.24**
JA3	**10**	40.11 ± 2.30**	74.28 ± 2.09**
	20	45.02 ± 2.09***	62.03 ± 2.11**

All values are expressed as mean ± SEM, *n* = *8*. One way ANOVA after which Dunnett's post hoc multiple comparison test to determine the values of P. ^!!!^P˂0.001 as comparison of diabetic control group *vs* control group. *P˂0.05, **P˂0.01 and ***P˂0.001 as comparison of diabetic control group *vs* test samples and glibenclamide treated groups, using one way ANOVA followed by Dunnet comparison.

The article "Chalcones: The flavonoid derivatives synthesis, characterization, their antioxidant and in vitro/in vivo antidiabetic potentials" was published in 2023. Journal: Heliyon.

#### 3.7.1 Effects on cholesterol

The recorded blood cholesterol level of the control group was 87.71 mg/dl whereas for diabetic group it was 182.79 mg/dl. For the compound treated groups a lowering effect on cholesterol level was observed which signifies antilipidemic effects of the compounds. The group treated with **JA1** with a dose of 10 mg/kg b. w lowered the blood cholesterol level to 137.33 md/dl whereas the same compound in at high dose of 20 mg/kg b. w brought this level to 120.71 mg/dl. **JA2** at the tested low and high doses lowered the CH level to 145.39 and 134.29 mg/dl respectively. For **JA3** treated group the recorded CH level was 130.15 mg/dl and 110.09 mg/dl for low and high tested doses respectively whereas the group administered with standard drug the CH level recorded was 89.93 mg/dl (Table 7). Among the tested compounds **JA3** has shown significant activities. The effect of compound on total CH and TG have been presented in Fig. 6.

**Fig. 6:** The synthesized chalcones effect the level of TCH and TG.

**Fig. 7:** Effect of synthesized chalcones on HDL level.

#### 3.7.2 Effects on TG

The level of TG rises with high intakes of oil and in diabetes mellitus. From Tables 7 and it is evident that the TG level recorded for normal control group was 82.66 mg/dl whereas it was almost two folds in diabetic group animals (165.39 mg/dl). The group treated with **JA1** at doses of 10 and 20 mg/kg body weight brought improvement in TG level to 136.11 mg/dl and 121.15 mg/dl respectively. **JA2** administration with the mentioned doses respectively brought its level to 138.70 mg/dl and 120.38 mg/dl whereas **JA3** was found to be the most potent compound which brought further improvements in TG levels to 127.86 mg/dl and 101.49 mg/dl. For standard group the level recorded was 84.05 mg/dl.

#### 3.7.3 Effects on HDL

Normally with diabetes the level of HDL falls down that is used as index of DX. As can be seen from Table 7, the HDL level for normal control group is 50.19 mg/dl which has dropped with STZ injection in diabetic group animals to 20.89 mg/dl. When the STZ diabetic rats were given the tested doses respectively, an improvement in this level to 36.71 mg/dl and 39.62 mg/dl after treatment with **JA1** was brought about, showing a mild effect in ameliorating the diseased conditions. **JA2** treated animals at tested low and high doses has improved the HDL level to 33.81 mg/dl and 35.94 mg/dl as recorded respectively. The **JA3** has again produced pronounce effect at tested doses as 40.11 mg/dl and 45.02 mg/dl respectively indicating to a potent antidiabetic agent. The standard drug have brought it to 48.10 mg/dl HDL being a standard drug (Table 8).

The article "Chalcones: The flavonoid derivatives synthesis, characterization, their antioxidant and in vitro/in vivo antidiabetic potentials" was published in 2023. Journal: Heliyon.

#### 3.7.4 Effects on LDL

The LDL level rises in diabetes which is clear from its values in normal control and diabatic control groups (36.87 mg/dl and 133.69 mg/dl respectively). The **JA1** treatment at doses of 10 and 20 mg/kg b. w respectively have brought this level to 82.83 md/dl and 77.28 mg/dl indicating the hypolipidemic effect of this compound. For the same doses, **JA2** have brought about a decrease with values of 90.87 mg/dl and 78.31 mg/dl respectively. For group treated with **JA3** at the tested doses the ameliorating effect was more pronounced with values 74.28 mg/dl and 62.03 mg/dl. For the Glibenclamide group the level was found to be 39.88 mg/dl. Among the tested compounds **JA3** was found to be the most potent compound to be used as diabetic drug.

### 3.8 Effects on liver related biochemical parameters

Table 8 indicates that there is a significant increase in the level of alanine phosphatase (ALP), Serum glutamic pyruvic transaminase (SGPT), serum glutamic-oxaloacetic transaminase (SGOT) and Serum creatinine levels in the diabetic animals as compared to normal control group animals. Administration of the **JA1**, **JA2** and **JA3** at doses of 10 and 20 mg/kg b. w has profoundly lowered the level of ALP, SGPT, SGOT and serum creatinine in the STZ diabetic group animals in various groups. The insulin level in diabetic rats was lowered as compared to the level recorded for normal control group. The observed increase in insulin level was brought near to normal by tested compounds as described below.

#### 3.8.1 Effects on ALP

The recorded value of ALP in the normal control group was 138.71 IU whereas for diabetic group the recorded vale was. 281.44 IU. **JA1** has dropped its high level brought about by STZ injection to 180.75 and 166.88 IU for 10 and 20 mg/kg b. w doses respectively. In **JA2** treated group, the ALP level for the mentioned doses were recorded as 187.59 and 167.87 IU**.** The **JA3** at the doses applied brough the ALP level to 168.62 and 153.90 IU. The Glibenclamide brough ALP level to 141.29 IU. **JA3** was considered to be the most effective compound than the other two. The overall results are summarized in Fig. 8.

The article "Chalcones: The flavonoid derivatives synthesis, characterization, their antioxidant and in vitro/in vivo antidiabetic potentials" was published in 2023. Journal: Heliyon.

**Fig. 8:** Effect of synthesized chalcones on ALP level.

#### 3.8.2 Effects on SGPT

The SGPT level was 21.09 IU for control group whereas for diabetic group it was 61.96 IU. **JA1** exhibited lowering effect on SGPT level for the tested high and low doses (38.08 and 43.61 IU respectively; as shown in Fig. 9). **JA2** and **JA3** also exhibited lowering effects of SGPT level administered in two doses mentioned with values 45.10 and 38.18 IU/37.19 and 30.87 IU whereas control being the standard drug has lowered the level to 23.03 IU. From the decreased level (SGPT) recorded for compounds under study, **JA3** was found to be more potent rather the other two compounds.

**Fig. 9:** Effect of synthesized chalcones on SGPT and SGOT level.

#### 3.8.3 Effects on SGOT

The observed level of SGOT (Fig. 8) for control group animals was 20.97 IU whereas after getting diabetes this level increased to 43.86 IU in animals of diabetic group. The groups after getting the **JA1** at doses of 10 and 20 mg/kg b. w lowered the SGOT level to 30.37 28.81 IU. **JA2** has also a lowering effect on the level of SGOT as recorded for the mentioned doses as 32.62 and 31.37 IU corresponding whereas the drop in its level recorded for **JA3** was 25.87 and 23.95 IU which more pronounced among the tested compounds. The Glibenclamide has lowered the level to 22.41 IU.

#### 3.8.4 Effects on serum creatinine

The effect of synthesized compounds on creatinine level is summarized in Table 9. For normal control and diabetic group, the creatinine level recorded was 1.03 mg/dl and 2.96 mg/dl respectively, indicating that with diabetes its level rises that could be used as marker while assessing diabetes in human. **JA1** treatment at tested doses brought the level to 1.31 and 1.20 mg/dl respectively, showing the compound's potency to be used as antidiabetic drug. Similarly, groups treated with **JA2** at the tested doses have brought its level to 1.39 and 1.26 mg/dl whereas a more pronounced effect was observed with **JA3** (1.19 and 1.07 mg/dl respectively for tested low and high doses). Glibenclamide with a dose of 0.5 mg/kg b. w lowered creatinine level to 0.93 mg/kg being the available drug in market.

**Table 9:** Effects on liver biochemical parameters.

Groups/dose mg/kg		ALP (IU)	SGPT (IU)	SGOT (IU)	Serum creatinine (mg/dL)	Insulin level (μU/mL)
**Normal control**		138.71 ± 3.50	21.09 ± 1.81	20.97 ± 1.33	1.03 ± 0.39	18.01 ± 1.41
**Diabetic control**		281.44 ± 4.32^!!!^	61.96 ± 2.03^!!!^	43.86 ± 1.90^!!!^	2.69 ± 0.55^!!!^	6.05 ± 0.87
**Glibenclamide (0.5)**		141.29 ± 3.86***	23.03 ± 1.91***	22.41 ± 1.66***	0.93 ± 0.21***	17.03 ± 1.31***
**JA1**	**10**	180.75 ± 4.75*	43.61 ± 3.01*	30.37 ± 2.09**	1.31 ± 0.60*	12.88 ± 1.21*
	**20**	166.88 ± 3.87*	38.08 ± 2.39*	28.81 ± 2.11**	1.20 ± 0.43**	13.59 ± 1.76**
**JA2**	**10**	187.59 ± 4.34*	45.10 ± 2.31*	32.62 ± 2.01*	1.39 ± 0.51*	12.17 ± 1.22*
	**20**	167.87 ± 4.53**	38.18 ± 2.52*	31.37 ± 2.31*	1.26 ± 0.33*	12.84 ± 1.30*
**JA3**	**10**	168.62 ± 4.04**	37.19 ± 2.46**	25.87 ± 2.20**	1.19 ± 0.39**	14.02 ± 1.59**
	**20**	153.90 ± 4.21***	30.87 ± 2.02***	23.95 ± 1.98***	1.07 ± 0.28**	14.68 ± 1.62**

All values are expressed as mean ± SEM, *n* = *8*. One way ANOVA after which Dunnett's post hoc multiple comparison test to determine the values of P. ^!!!^P˂0.001 as comparison of diabetic control group *vs* control group. *P˂0.05, **P˂0.01 and ***P˂0.001 as comparison of diabetic control group *vs* test samples and glibenclamide treated groups, using one way ANOVA followed by Dunnet comparison.

The article "Chalcones: The flavonoid derivatives synthesis, characterization, their antioxidant and in vitro/in vivo antidiabetic potentials" was published in 2023. Journal: Heliyon.

#### 3.8.5 Effects on insulin level

It is an established fact that with diabetes the insulin level drops down as is clear from comparison of normal and diabetic control group values (18.01 μU/mL and 6.05 μU/mL respectively). The chalcone **JA1** with a dose of 10 mg/kg b. w enhanced the level of insulin to 12.88 μU/mL whereas at a high dose its level was further enhanced to 13.59 μU/mL. Same enhancing effect on insulin level was recorded for **JA2** and **JA3** at the tested doses (12.17/12.84 μU/mL and 14.02/14.68 μU/mL respectively). Comparatively the **JA3** was more potent as their values were near to Glibenclamide (17.03 μU/mL), the standard.

## 4 Conclusions

Diabetes mellitus is the third most prevalent agent of death causalities after cancer and heart attack. Scientists are therefore, struggling to explore antidiabetic agents both from plants and synthetic origin. The present study was aimed to synthesize, characterize and evaluate the chalcones; the flavonoids as antioxidant and antidiabetic agents. The desired compounds were synthesized from aromatic aldehyde and acetophenone. Spectroscopic techniques were used to identify and confirm their formation which were then evaluated for their antioxidant and antidiabetic potential in *in-vitro*. The compounds were evaluated for antidiabetic and toxicological potential in rat's model. The **JA3** was found to be the most potent compounds with low values of IC_50_ against DPPH free radical and alpha glucosidase whereas the effects on blood glucose level in rats at the tested dose was also appreciable. The disturbance brough about by diabetes induce in rats in the form blood biochemical parameters was normalized by **JA3** almost similar in response to standard acarbose. Thus, **JA3** may further be subjected to *in vivo* evaluation in other animal models to extend and ensure its use as antioxidant and antidiabetic drug in human in near future. It is also suggested to evaluate the pre-clinical safety profile in animal model for *in-vivo* acute, sub-chronic, and chronic toxicity on vital organs.

The article "Chalcones: The flavonoid derivatives synthesis, characterization, their antioxidant and in vitro/in vivo antidiabetic potentials" was published in 2023. Journal: Heliyon.

## 5 Data availability statement

No data was used for the research described in the article.

## Funding statement

Princess Nourah bint Abdulrahman University Researchers Supporting Project (number PNURSP2023R33), Princess Nourah bint Abdulrahman University, Riyadh, Saudi Arabia.

## CRediT authorship contribution statement

**Jalal Uddin:** Writing – original draft, Methodology, Formal analysis. **Syed Wadood Ali Shah:** Supervision, Methodology, Conceptualization. **Muhammad Zahoor:** Writing – review & editing, Supervision, Project administration, Conceptualization. **Riaz Ullah:** Resources, Investigation, Funding acquisition, Formal analysis, Data curation. **Amal Alotaibi:** Writing – original draft, Resources, Funding acquisition, Formal analysis, Conceptualization.

## Declaration of competing interest

The authors declare that they have no known competing financial interests or personal relationships that could have appeared to influence the work reported in this paper.
